# The Relationship between Gestational Newborn Weight Loss and Hospitalization in the First Week after Birth

**DOI:** 10.1155/2022/9871177

**Published:** 2022-08-08

**Authors:** Linxiao Qiao, Haiyan Zhang, Yufeng Yuan, Wenying Zhu, Jing Yuan, Yuanyuan Hu, Hongli Zhu

**Affiliations:** ^1^Department of Pediatrics, The First People's Hospital of Kunshan Affiliated to Jiangsu University, China; ^2^Department of Pediatrics, Kunshan Maternity and Children's Health Care Hospital, Kunshan, China; ^3^Department of Pediatrics, Huai'an Maternal and Child Health Care Center, Huaian, Jiangsu, China

## Abstract

**Objective:**

To investigate the association of weight loss daily of term infants with hospitalization in the first week after birth.

**Methods:**

This prospective cohort study was conducted among 1865 infants from May 2020 to June 2021, born in the Department of Obstetrics, Kunshan's First People's Hospital Affiliated to Jiangsu University and Huai'an Maternal and Child Health Care Center. The infants' weight was collected daily in the hospital, and the weight loss was calculated daily. According to the weight loss daily, the infants were divided into 3 groups. Group A: the weight loss per day was less than 2% of birth weight, and the total weight loss was less than 10%. Group B: the weight loss per day was between 2 and 4% of the birth weight, and the total weight loss was less than 10%. Group C: the weight loss per day was more than 4% of the birth weight, or the total weight was more than 10%. The infants in group C were monitored carefully in the hospital or Outpatient Department (OPD) daily. The primary outcome was the incidence of hospitalization.

**Results:**

Of the 1865 term infants enrolled, 1052 were completed on the 7^th^ day (356 in group A, 513 in group B, and 183 in group C). There was no significant difference among the three groups of subjects in terms of infant data, including birth weight, gender, Apgar scores, and gestational age. The number of C-sections and primiparas was substantially higher in groups C and B than in group A. The incidence of hospitalization in group C was significantly higher than that in group A and group B (30.6%, 12.1%, and 12.5%, respectively). The incidence of exclusive breastfeeding in group C was significantly lower than that in group A and group B (28.4%, 41%, and 38.4%, respectively). There was no significant difference between group A and group B in the incidence of hospitalization and exclusive breastfeeding. Most of the hospitalization was because of hyperbilirubinemia, and in group C, there were 2 babies because of dehydration fever and 3 because of hypoglycemia.

**Conclusions:**

The neonates whose weight loss daily after birth was more than 4% of the total weight loss of more than 10% had higher hospitalization rates.

## 1. Introduction

It is common for babies to experience losing weight in the first week after birth. The studies showed that the physiological neonatal weight loss in term infants is less than 10% of the birth weight [1, 2]. A substantial risk of severe health consequences, such as hyperbilirubinemia, hypernatremic dehydration, and hypoglycemia, is associated with excessive weight loss [3–6]. World Health Organization suggests losing 10% of birth weight in the first week of life as a threshold for further assessment [1]. The American Academy of Pediatrics recommends that >7% weight loss within the first 3 to 5 days is excessive for a healthy, full-term, breastfed infant (American Academy of Pediatrics and The American College of Obstetricians and Gynecologists, 2012). But there have no guidelines or appropriate growth charts for the babies in the first week after birth because of the lack of evidence-based data [7, 8].

And there is no suggestion about how much weight loss per day will be appropriate. Therefore, the present study was aimed at investigating how much weight loss per day will be suitable.

## 2. Research Methodology

### 2.1. Patients

This prospective cohort study was conducted among 1865 infants from May 2017 to July 2021 at the mother-infant unit, The First People's Hospital of Kunshan Affiliated to Jiangsu University and Huai'an Maternal and Child Health Care Center. The inclusion criteria were gestational age between 37 and 42 weeks infants. Exclusion criteria included (1) preterm infants, (2) postterm infants, (3) birth weight less than 2500 g, and (4) transfer to NICU within 24 h after birth. Ethical approval was obtained from the Research Ethical Committee of The First People's Hospital in Kunshan, Jiangsu University. Informed consent forms were signed and collected from the study's participants.

### 2.2. Groups

The infants' weight was collected daily in the hospital, and the weight loss was calculated daily. The sheets were collected. According to the weight loss daily, the infants were divided into 3 groups. Group A: the weight loss per day was less than 2% of birth weight, and the total weight loss was less than 10% (of birth weight). Group B: the weight loss per day was between 2 and 4% of the birth weight and the total weight loss less than 10%, the feeding was reassessed, and breastfeeding was instructed again. Group C: the weight loss per day was more than 4% of the birth weight, or the total weight was more than 10%; the situation of mother and infant was reassessed; and breastfeeding was instructed again. If the total weight loss of the infants in group A or group B was more than 10% of birth weight, the infants were included in group C. The infants needed strengthening feeding (including breastfeeding and supplement formula), and blood sugar and urine volume were monitored.

After discharge, the weight was recorded, the feeding was reassessed, and the nurse instructed breastfeeding by the telephone until seven days after birth. The infants in group C must be carefully monitored in the hospital or outpatient department daily. The infants in group C need the following: reassess the mother (including diet, ways of feeding, sleeping, pain, amount of breastfeeding, and medication) and baby (including vitals, urine output, blood sugar, dehydration, and signal of infection). Patients were withdrawn from the study if their parents were unwilling to participate. The infant-feeding policies and procedures at the Department of Obstetrics in the hospital comply with the WHO's Ten Steps to Successful Breastfeeding [9], which is considered the optimal standard of breastfeeding management in hospitals. Our routine practice is to reassess the mother and baby before the medical supplement formula unless the mother refuses to breastfeed.

### 2.3. Weight Measurement

All infants were routinely weighed at birth using SECA 335 weighing scale (Hamburg, Germany) (accurate to the nearest 5 g). Subsequent daily weights were obtained in the morning after the bath. The discharge of cesarean section babies was usually around 4-6 days, while the release of babies by vagina was normally 2 to 3 days. The family weighed (following hospital training guidelines) the babies daily after discharge until seven days after birth. The information was then gathered by the nurses and entered into the computer. The WHO's Ten Steps to Successful Breastfeeding were thoroughly explained to the nurses. When the total weight loss of the infants was more than 10% of birth weight, the infants in the hospital needed reassessment and strengthened feeding (including breastfeeding and supplement formula), blood sugar, hyperbilirubinemia, and urine volume were monitored. And if the infant was discharged, the baby and mother needed to see the doctor.

### 2.4. Observations and Measurement Parameters

We collected information on the mother's age, breastfeeding history, method of delivery, type of C-section (planned or unplanned), and pregnancy complications. Daily measurements were made of the infant's birth weight, sex, Apgar scores, gestational age, weight, and transcutaneous bilirubin. The incidence of hospitalization served as the primary outcome. The secondary endpoints were the duration it took to regain birth weight and the frequency of exclusive breastfeeding.

### 2.5. Statistical Analyses

Data were analyzed using SPSS (v.21.0) software for windows. Clinical characteristics of the three groups were expressed by mean values and standard deviations as mean ± SD (*x* ± *s*) and by rates and percentages. Between-group differences were analyzed using the *t*-test. The chi-square test examined differences in rates. *P* < 0.05 was considered to be statistically significant.

## 3. Results

### 3.1. General Characteristics of the Selected Groups

Of the 1865 term infants enrolled, 1823 completed the collected data on the first day. 1806 finished on the second day, 1765 on the third day, 1536 on the fourth day, 1354 on the fifth day, 1244 on the sixth day, and 1052 on the seventh day (356 in group A, 513 in group B, and 183 in the group C) (Figure 1). There was no significant difference among the three groups of subjects in terms of infant data included birth weight, gender, Apgar scores, and gestational age (Table 1). There was a significantly higher number of C-sections and primipara in group C and group B than in group A.

In the study, the incidence of hospitalization in group C was significantly higher than that in group A and group B (30.6%, 12.1%, and 12.5%, respectively). The incidence of exclusive breastfeeding in group C was significantly lower than that in group A and group B (28.4%, 41%, and 38.4%, respectively). There was no significant difference between group A and group B in the incidence of hospitalization and exclusive breastfeeding (Table 1). Most of the hospitalization was because of hyperbilirubinemia, and in group C, there were 2 babies because of dehydration fever and 3 because of hypoglycemia (Table 2).

## 4. Discussion

The current study showed that the high risk of hospitalization increased and the rate of exclusive breastfeeding decreased when the weight loss of term infants after birth was more than 4 percent per day or total weight loss of more than 10%, which was more easily occurred in the babies of primipara and C-section mothers.

On the 7^th^ day after birth, 1052 newborns were included in the study (356 in group A, 513 in group B, and 183 in group C). It was a staggering rate of weight loss of more than 4% each day or more than 10% overall (17.4%). Similarly, Bertini et al.'s study revealed no infants dropped more than 10% of their body weight [10]. The high incidence in our study may be 2 reasons. One was the high C-section in our Department. The other reason was the WHO's Ten Steps to Successful Breastfeeding were not fulfilled well [8]. There must be more training, education, and compliance about breastfeeding [11]. And social reasons, C-sections need to be controlled. Group C had a much more significant proportion of primipara than groups A and B. It might be because first-time mothers are more likely to feel anxious about breastfeeding, think their milk supply is not enough, and ask for supplements for their babies [12]. So in infants, especially primiparous and C-section mothers, there need more attention, monitoring, and breastfeeding [13, 14].

The incidence of hospitalization in group C was significantly higher than that in group A and group B (30.6%, 12.1%, and 12.5%, respectively). Most of the hospitalization was because of hyperbilirubinemia, and in group C, there were 2 babies because of dehydration fever and 3 because of hypoglycemia. A study showed that increasing breastfeeding frequency and accelerated weight gain could reduce the severity of neonatal hyperbilirubinemia [6]. So in the first week after birth, the infants needed breastfeeding frequency. If the mother had insufficient breastfeeding, there needed more direction; then, a medical supplement was required [11]. When the weight loss was more than 4% daily or total weight loss was more than 10%, the mother was reassessed; if there was not enough breastfeeding, a medical supplement was needed. Otherwise, the risk of hospitalization may be increased.

The incidence of exclusive breastfeeding in group C was significantly lower than that in group A and group B (28.4%, 41%, and 38.4%, respectively). The rate of exclusive breastfeeding on the first weekend was lower than in the studies. We thought the WHO's Ten Steps to Successful Breastfeeding were not fulfilled well. And the rate in group C was the lowest. The other reason was the high hospitalization made breastfeeding difficult and the mother more anxious [15]. It is necessary to highlight the study's limitations. There was a large percentage of excluded data and fewer members of group C than of groups A and B, which increased the possibility of bias. Therefore, more research is required to validate the present study findings.

## 5. Conclusion

The current study concluded that newborns with more than 4% daily weight decline and more than 10% overall weight loss experienced a greater risk of hospitalization rates.

## Figures and Tables

**Figure 1:** General characteristics of the selected groups.

**Table 1:** Clinical characteristics and outcomes of the groups chosen.

	Group A (*n* = 356)	Group B (*n* = 513)	Group C (*n* = 183)	*P* ^A-B^ value	*P* ^B-C^ value	*P* ^A-C^ value
Gender (M/F)	182/174	265/248	94/89			
Gestational age (w)	39.6 ± 0.8	38.4 ± 1.1	38.6 ± 1.3	0.432	0.856	0.921
Birth weight (g)	3423 ± 392	3225 ± 202	3375 ± 249	0.435	0.754	0.667
Apgar score	8.5 ± 1.2	8.8 ± 1.4	8.7 ± 0.9	0.573	0.748	0.584
Maternal age	29.3 ± 3.6	30.2 ± 4.2	28.7 ± 5.3	0.441	0.754	0.332
Number of C-section (%)	121 (34)	186 (36.3)	89 (48.6)	0.491	0.033^∗^	0.001^∗^
Number of primipara	187 (52.5)	276 (53.8)	122 (66.7)	0.7114	0.0025^∗^	0.0017^∗^
Incidence of hospitalization	43 (12.1)	64 (12.5)	56 (30.6)	0.8610	<0.001^∗^	<0.001^∗^
Incidence of exclusive breastfeeding	146 (41)	197 (38.4)	52 (28.4)	0.4389	0.0155^∗^	0.041^∗^

*P* ^A-B^: group A versus group B; *P*^B-C^: group B versus group C; *P*^A-C^: group A versus group C.

**Table 2:** Reasons for hospitalization of the three groups.

	Group A (*n* = 356)	Group B (*n* = 513)	Group C (*n* = 183)
Incidence of hospitalization	43 (12.1)	64 (12.5)	56 (30.6)
Number of hyperbilirubinemia	26	37	39
Number of hypoglycemia	0	1	3
Number of dehydration fever	0	0	2
Number of infection	5	12	8
Other diseases	12	14	4

## Data Availability

Data will be provided upon request to the authors.

## References

[1] Flaherman V. J., Schaefer E. W., Kuzniewicz M. W., Li S. X., Walsh E. M., Paul I. M. (2015). Early weight loss nomograms for exclusively breastfed newborns. *Pediatrics*.

[2] Chantry C. J., Nommsen-Rivers L. A., Peerson J. M., Cohen R. J., Dewey K. G. (2011). Excess weight loss in first-born breastfed newborns relates to maternal intrapartum fluid balance. *Pediatrics*.

[3] American Academy of Pediatrics (2004). Management of hyperbilirubinemia in the newborn infant 35 or more weeks of gestation. *Pediatrics*.

[4] Lambrinou C. P., Karaglani E., Manios Y. (2019). Breastfeeding and postpartum weight loss. *Current Opinion in Clinical Nutrition and Metabolic Care*.

[5] Mulder P. J., Johnson T. S., Baker L. C. (2010). Excessive weight loss in breastfed infants during the postpartum hospitalization. *Journal of Obstetric, Gynecologic, and Neonatal Nursing*.

[6] Hassan B., Zakerihamidi M. (2018). The correlation between frequency and duration of breastfeeding and the severity of neonatal hyperbilirubinemia. *The Journal of Maternal-Fetal & Neonatal Medicine*.

[7] Fonseca M. J., Severo M., Santos A. C. (2015). A new approach to estimating weight change and its reference intervals during the first 96 hours of life. *Acta Paediatrica*.

[8] Fewtrell M. S., Morgan J. B., Duggan C. (2007). Optimal duration of exclusive breastfeeding: what is the evidence to support current recommendations?. *The American Journal of Clinical Nutrition*.

[9] World Health Organization, Division of Child Health and Development (1998). *Evidence for the ten steps to successful breastfeeding*.

[10] Bertini G., Breschi R., Dani C. (2015). Physiological weight loss chart helps to identify high-risk infants who need breastfeeding support. *Acta Paediatrica*.

[11] Academy of Breastfeeding Medicine Protocol Committee (2009). ABM clinical protocol #3: hospital guidelines for the use of supplementary feedings in the healthy term breastfed neonate, revised 2009. *Breastfeeding Medicine*.

[12] Deng X., McLaren M. (2018). Using 24-hour weight as reference for weight loss calculation reduces supplementation and promotes exclusive breastfeeding in infants born by cesarean section. *Breastfeeding Medicine*.

[13] Victora C. G., Bahl R., Barros A. J. (2016). Breastfeeding in the 21st century: epidemiology, mechanisms, and lifelong effect. *Lancet*.

[14] Gartner L. M., Morton J., Lawrence R. A. (2005). Breastfeeding and the use of human milk. *Pediatrics*.

[15] Salas A. A., Salazar J., Burgoa C. V., De-Villegas C. A., Quevedo V., Soliz A. (2009). Significant weight loss in breastfed term infants readmitted for hyperbilirubinemia. *BMC Pediatrics*.

